The article "Targeting Tumor Microenvironment by Metal Peroxide Nanoparticles in Cancer Therapy" was published in 2022. Journal: Bioinorg Chem Appl.

# Targeting Tumor Microenvironment by Metal Peroxide Nanoparticles in Cancer Therapy

**DOI:** 10.1155/2022/5041399

**Published:** 2022-12-16

**Authors:** Simon Ngigi Mbugua

**Affiliations:** Department of Chemistry, Kisii University, P.O. Box 408-40200, Kisii, Kenya

## Abstract

Solid tumors have a unique tumor microenvironment (TME), which includes hypoxia, low acidity, and high hydrogen peroxide and glutathione (GSH) levels, among others. These unique factors, which offer favourable microenvironments and nourishment for tumor development and spread, also serve as a gateway for specific and successful cancer therapies. A good example is metal peroxide structures which have been synthesized and utilized to enhance oxygen supply and they have shown great promise in the alleviation of hypoxia. In a hypoxic environment, certain oxygen-dependent treatments such as photodynamic therapy and radiotherapy fail to respond and therefore modulating the hypoxic tumor microenvironment has been found to enhance the antitumor impact of certain drugs. Under acidic environments, the hydrogen peroxide produced by the reaction of metal peroxides with water not only induces oxidative stress but also produces additional oxygen. This is achieved since hydrogen peroxide acts as a reactive substrate for molecules such as catalyse enzymes, alleviating tumor hypoxia observed in the tumor microenvironment. Metal ions released in the process can also offer distinct bioactivity in their own right. Metal peroxides used in anticancer therapy are a rapidly evolving field, and there is good evidence that they are a good option for regulating the tumor microenvironment in cancer therapy. In this regard, the synthesis and mechanisms behind the successful application of metal peroxides to specifically target the tumor microenvironment are highlighted in this review. Various characteristics of TME such as angiogenesis, inflammation, hypoxia, acidity levels, and metal ion homeostasis are addressed in this regard, together with certain forms of synergistic combination treatments.

## 1. Introduction

Cancer has risen to become one of the major threats to human health, and it is reported to have caused approximately 10 million deaths globally in 2020 alone, according to data available on the WHO website (https://www.who.int/news-room/fact-sheets/detail/cancer). This accounts for nearly one in six deaths, making cancer the biggest cause of mortality globally, with breast, lung, colon, rectum, and prostate cancers being the most prevalent types of cancer.

According to the American Cancer Society, in the United States of America alone, an estimated 609,000 people died of cancer in the year 2021 with lung and colon cancers being the most prevalent among both men and women. In the same period, 1,898,160 new cases of cancer were reported (Figure 1) [1].

From such grim statistics, the advancement and development of new approaches to combat this disease are critical. With the advancement of technology in scientific research, a number of unique cancer treatment approaches have been developed. These include photodynamic therapy (PDT), chemodynamic therapy (CDT), photothermal therapy, and nanoparticles, among others, which have been developed to complement the standard treatments which utilize chemotherapy and radiation [2].

Many technologies are now being investigated in clinical trials, and some have even been adopted in clinical practice. Targeted delivery of active drugs, delivery by nanoparticles, and targeting overexpressed proteins and antigens on tumor cell surfaces are a few of these methods [3]. The ability to treat cancer has advanced enormously over the past 70 years, from cytotoxic medications that shrink tumors but have serious systemic side effects, to targeted therapies that may kill cancer cells while sparing healthy organs. This article discusses some of the new approaches that target the tumor microenvironment (TME) by the use of metal peroxides to alter the oxygen levels in tumors [4, 5].

Many issues still need to be studied in order to further understand cancer therapy. Research is making significant efforts to find novel and efficient treatments that can lessen side effects. This has been the focus over the past ten years, where several research studies have concentrated on developing alternative therapies to reduce the negative effects of conventional medications [6, 7].

The departure from the cisplatin operation model, which employs the metal as the principal active centre of the therapy is a developing trend, even though the traditional chemotherapy approach using DNA as the set target continues to yield significant results. Most of the available and effective anticancer medications currently on the market are met with high toxicity levels [8, 9]. Cancer research may be considered as an area with significant unmet needs since cancers also acquire immunity against most medications [10–12].

Metal-based drug platforms for cancer therapy have been used for a long time and have been shown to perform well in the detection and treatment of illnesses, and they are critical in the early stages of therapeutic development. Chief among these are platinum-containing medications which are the most extensively studied and used as antitumor chemotherapy treatments [13–15]. They constitute one of the main triumphs in the field of application of medical bioinorganic chemistry. These drugs which include cisplatin, carboplatin, and oxaliplatin, all in the class of cell cycle nonspecific treatments, are being employed in disorders such as gynaecological and digestive system cancers [16, 17].

Their mechanism of action involves penetrating the nucleus of a cell and reacting with DNA molecules to produce platinum-DNA complexes, which distort DNA structure and prevent replication and transcription [18, 19]. Antitumor medicines containing platinum, on the other hand, have drawbacks such as limited bioavailability, high systemic toxicity, resistance, and limited selectivity for cancerous cells [20, 21].

In particular, when platinum medications and proteins are combined in the blood, the reaction inactivates most of these drugs before they reach the desired targets [22]. This results in severe side effects as well as decreased bioavailability, thereby reducing the efficacy of these treatments [21]. Furthermore, typical platinum medications primarily target the genome, which in some cases is easily repaired by cancer cells. This raises the susceptibility of these cells to platinum drug resistance [11, 23].

In the physiological environment, metal ions are known to play key roles in a variety of important cellular metabolic pathways including material movement into and out of the cell across the cell membrane, energy production, and transmission of information, among others [24, 25]. When these ions are not properly distributed or absorbed in cells, this can obstruct the aforementioned processes, resulting in permanent cellular injury, or the activation of metabolic responses which may lead to apoptosis [26, 27].

Metal peroxides have attracted particular research interest in biology and medicine due to their peculiar chemical reactions, associated reaction products, and particular biochemical effects of the released metal ions [28, 29]. Recently, versatile metal peroxide nanoparticles including CuO_2_, CaO_2_, MgO_2_, ZnO_2_, BaO_2_, and TiOx have been developed for therapeutic applications [30–32]. These include areas of cancer treatment, bacterial infection prevention, and tissue regeneration, where they have received substantial research attention [33, 34].

For many years, the logical design of drug targeting techniques has been explored, and flexible targeting protocols have been suggested to increase targeting effectiveness [35, 36]. However, targeting strategies are still far from ideal. The investigation of disease-specific therapy by inducing chemical reactions in situ has sparked intense study interest. Numerous nanoparticles that can initiate favourable chemical processes for the treatment of diseases are now being developed, either as nanocatalysts or nanoreactants [37, 38]. Since these nanomedicines are designed to respond to specific disease microenvironments, they are expected to improve drug targeting and therefore efficacy, at the same time reducing undesirable side effects.

Consisting primarily of metal ions and peroxo groups, metal peroxides may combine with water to form hydrogen peroxide and release metal ions in the process [34]. Numerous biological applications can benefit from the postgenerated hydrogen peroxide. For instance, in catalytic medicine, hydrogen peroxide can function as the reactant in a Fenton-like enzymatic reaction to produce large amounts of extremely harmful hydroxyl radicals [39]. The therapeutic effectiveness of procedures that involve oxygen, such as photodynamic treatment (PDT) and radiotherapy, can also be increased by the self-decomposition of hydrogen peroxide to create oxygen [40, 41].

The metal-ion component of metal peroxides takes part in a variety of biological processes, such as biochemical reactions and the process of tissue regeneration [42, 43]. On this basis, metal peroxide-based nanoparticles serve as nascent nanosystem with distinct intrinsic physicochemical characteristics, reactive aspects, and bioactivities for fulfilling diverse requirements of biological applications. Copper peroxide (CuO_2_), calcium peroxide (CaO_2_), magnesium peroxide (MgO_2_), zinc peroxide (ZnO_2_), barium peroxide (BaO_2_), and titanium peroxide (TiOx) are some of the metal peroxide nanosystems which have attracted interest in this area. As shown in Figure 2, they have been extensively investigated in several biomedical fields, including catalytic nanomedicine, based on their reactivity for hydrogen peroxide and oxygen generation and metal ion-based bioactivity [44–46].

## 2. Targeting the Tumor Microenvironment

Without a crucial interaction between cancerous cells and their immediate environment, the malignant characteristics of cancer cells cannot appear. Cancer growth is actively aided by the tumor infiltrate, which is made up of immune cells, angiogenic vasculature, lymphatic cells, and cancer-associated fibroblastic cells [47]. The capacity to alter these conditions is a crucial trait that allows tumor cells to develop some of the characteristic abilities required for tumor development and metastatic spread. Therefore, it has become essential in the area of cancer therapy to target the tumor microenvironment as a viable frontier in cancer treatment.

The notion of a complex tumor environment that promotes tumor growth and metastatic dispersion has replaced the tumor cell-centered perspective of cancer development as a result of the realization of the TME's crucial role in the genesis and progression of cancer [48]. As a result, new TME targets have been found that may assist, guide, and enhance the effects of numerous cancer medicines. The functioning of the tumor microenvironment (TME) dictates its fundamental and essential role in tumor morphology and physiology [49].

Numerous immune and nonimmune cell types may be detected inside the TME infrastructure, and together with the numerous substances they emit, these cells help to create an intratumoral milieu that is chronically inflammatory, immunosuppressive, and proangiogenic [50]. In these conditions, cancer cells can adapt and develop with a considerably lower chance of being found and eliminated by host immune surveillance. The number of biological molecules and mechanistic pathways that might be targeted for cancer treatment grows as our understanding of the TME expands. Here, a few of these particular microenvironments shown in Figure 3 are discussed.

### 2.1. Targeting Angiogenesis through Anti-VEGF Drugs

Proangiogenic and antiangiogenic factors generated by both malignant and nonmalignant cells tightly regulate the complicated process of vascularization in tumors through a number of signalling channels [51]. When proangiogenic factors are more prevalent, angiogenesis, sometimes referred to as the “angiogenic switch,” is activated [52]. The main proangiogenic factor in endothelial cell activation is the vascular endothelial growth factor-A (VEGF-A), although numerous other growth factors, including fibroblast growth factor (FGF), platelet-derived growth factor (PDGF), and endothelial growth factor (EGF), are also proangiogenic [53]. The tumor vasculature with a deficit in pericytes and perivascular cells, as well as an increased permeability, leads to a leaky vascular system [54, 55]. This is in contrast to normal vasculature, which is characterized by an organized formation of mature endothelial cells covered with pericytes [56].

In vasculogenesis, the newly created blood vessels' ability to supply oxygen and nutrients contributes to tumor growth and proliferation [52]. Therefore, targeting angiogenesis is a potential option for therapeutic intervention in cancer treatment. Antiangiogenic medications which cause leaky vasculature have now been the subject of numerous clinical studies globally [57]. When used in conjunction with traditional chemotherapy treatments, the anti-VEGF antibody bevacizumab improves overall survival in patients with metastatic colorectal cancer, nonsmall cell lung cancer, and breast cancer [58, 59].

### 2.2. Targeting Inflammation through Anti-Inflammatory Drugs

Studies recognise persistent inflammation as a key player in the development of cancer [60]. Laboratory studies suggest that the presence of active chronic innate immune cell types, such as neutrophils, macrophages, and mast cells (MCs) promote tumorigenesis [61]. This is performed through tissue remodelling, instigation of angiogenesis, and uncontrolled cell proliferation, leading to the growth and advancement of malignant cells into ectopic tissue [61]. In this regard, a number of anti-inflammatory medications, including cyclooxygenase 2 inhibitors have been tested for colorectal and chemotherapy-resistant breast cancer [62, 63]. Nonsteroidal anti-inflammatory drugs are reported for breast, colorectal, and prostate cancer treatment [64]. Anti-inflammatory steroid drugs such as dexamethasone used for the treatment of brain tumors, have been found to lower tumor incidence and slow down tumor progression and lower overall mortality rates [65].

### 2.3. Targeting the Noncellular Tumor Microenvironment

In addition to extracellular matrix (ECM) molecules, the noncellular environment also consists of physical and chemical elements including pH, oxygen tension, interstitial pressure, and fluid flow [66]. Therefore, any alterations in ECM in the context of the tumor environment will have an impact on cancer cell activity. The ECM is increasingly understood to be a dynamic component of the tumor microenvironment rather than a static structure that only preserves tissue shape. Cell proliferation, migration, angiogenesis, and cancer metastasis are all known to be regulated by ECM components and their metabolites [67, 68].

The ability of the tumor microenvironment to support cancer cell proliferation, migration, and invasion, as well as to affect inflammatory responses and lymphangiogenesis, can be significantly impacted by changes in ECM degradation such as density and stiffness [69]. A deeper comprehension of this complex ecosystem will be necessary to enhance cancer therapy due to the complexity of tumor cell-host cell interactions and cell-ECM interactions inside a tumor. It seems improbable that focusing on a specific molecular pathway or kind of cell would result in effective anticancer treatments and prevent the development of drug resistance. To achieve long-term effectiveness, it is necessary to combine conventional “cell-centred” chemotherapies and radiation therapies with strategies that target the no-cellular tumor microenvironment.

### 2.4. Targeting Hypoxia

One of the main characteristics that distinguish cancer cells from normal cells is their uncontrolled proliferative behaviour, which is partly caused by abnormal vasculature [70]. The oxygen level in places with solid tumors decreases as a result of the cancer cells' fast oxygen consumption. The fast proliferating cells result in a significant diffusion distance for oxygen, from the network of blood vessels, and the cancer cells. The result is a highly hypoxic scenario as a result of the tumor's lack of oxygenated blood, which encourages the growth of cells that turns tumorous [71]. Additionally, hypoxic circumstances encourage cancer cells to switch from oxidative phosphorylation to anaerobic glycolysis, which naturally causes lactic acid to accumulate and lower extracellular pH in the tumor microenvironment [72, 73].

Additionally, tumor-associated and/or therapy-induced anaemia reduces the blood's ability to carry oxygen, which results in hypoxia in tumor areas [74]. Poor prognosis, radiotherapy/chemotherapy resistance, and tumor metastasis are all linked to hypoxia [75]. Tumor cells can adapt to hypoxic conditions by producing erythropoietin (EPO), switching from aerobic to anaerobic metabolism, downregulating DNA repair pathways, enlisting the assistance of stromal cells, and upregulating protooncogenes as well as hypoxia-inducible factor (HIF) 1 and HIF 2 [76]. Therapeutic medicines are frequently created as low-toxicity prodrugs in normoxic environments and are then selectively activated in hypoxic tumor regions to address hypoxia in TME [77].

The hypoxia-activated prodrug AQ4N ((1,4-bis((2-(dimethylamino-N-oxide)ethyl)amino)5,8-dihydroxy-anthracene-9,10-dione), also known as banoxantrone, is transformed into AQ4, a strong inhibitor of topoisomerase II, in hypoxic environments, and treat solid malignancies including bronchoalveolar lung carcinoma and ovarian cancer [78]. Hemeproteins transform AQ4 from the aliphatic N-oxide prodrug by two successive 2e reductions. Under hypoxic circumstances, hypoxia-activated prodrugs called enamine N-oxides can release small molecules through selective bioreductive two-electron bioreduction processes [79]. The resultant iminium ion, which is unsaturated, is easily reactive with biological nucleophiles [80].

The reaction scheme in Figure 4 shows the mechanism of action for the AQ4N and enamine N-oxide prodrugs.

Tirapazamine (TPZ), another hypoxia cell toxin, selectively shows cytotoxic effects under an hypoxic environment [81]. Its mode of action is based on the process where several intracellular reductases catalyse TPZ to generate a radical by adding an electron [82]. In an hypoxic environment, this highly reactive TPZ radical can result in DNA single- or double-strand breaks [83]. The TPZ radical's cytotoxicity is quickly reduced when it is oxidized back to its harmless parent under aerobic circumstances [84]. Under hypoxic conditions, the metabolism of TPZ leads to the loss of a water molecule to generate the benzotriazinyl (BTZ) radical, which also leads to DNA damage as illustrated by the reaction mechanism in Figure 5.

### 2.5. Targeting the Acidic TME

Normal tissues have an extracellular pH of 7.4, but the pH in TME is substantially lower (6.7–7.1). There are several processes through which tumors develop an acidic pH. As discussed earlier, tumor cells in a hypoxic environment primarily employ aerobic glycolysis as an energy metabolism process [73]. This results in increased production of lactic acid and H^+^, which are then released in the tumor microenvironment (TME) by passive diffusion and active membrane-based ion transport [85]. Tumor cells have greatly elevated levels of the H + -ATPases, Na^+^-H^+^ exchanger NHE1, and monocarboxylate-H^+^ efflux cotransporters MCT1 and MCT4, and these factors all contribute to H+ efflux [86]. Additionally, the preservation of low pH in TME is also aided by carbonic anhydrase 9 (CA9), which is overexpressed in several cancer types [87].

To address acidity in TME, several researchers have reported that proton pump inhibitors may slow the growth of hepatoblastoma and oesophageal adenocarcinoma [88–90]. Proton pump inhibitors, such as omeprazole, esomeprazole, rabeprazole, pantoprazole, or lansoprazole, significantly slow the growth and development of neoplasms in individuals with Barrett's oesophagus [91]. Bafilomycin A1, a proton pump inhibitor of the vacuolar type, has demonstrated viability to induce apoptosis in hepatoblastoma cells but not in healthy cells, suggesting that it may be used as a cancer therapy [92].

## 3. Fenton-Reaction Approach

With a high level of tumor selectivity, Fenton reaction-based catalytic nanoparticles have become a unique tumor-therapeutic technique [93, 94]. Typically, Fenton compounds are used in oxidative treatment to cause a disproportionate reaction and transform tumors with overexpressed hydrogen peroxide into toxic hydroxyl radicals [95–97]. However, the therapeutic effectiveness of these catalytic-process-based nanotherapeutics is significantly constrained by the low intratumoral hydrogen peroxide level of around 100 *μ*m [98, 99]. The ability of metal peroxides to produce hydrogen peroxide opens up the idea of creating Fenton nanoagents for catalytic nanotherapeutics. Copper chloride, hydrogen peroxide, and sodium hydroxide have been used in an aqueous reaction system to easily create multifunctional copper peroxide (CuO_2_) nanodots [100, 101].

This procedure included polyvinylpyrrolidone (PVP) which not only regulates nanodot particle diameter but also supplies the surface functionalization necessary to ensure the excellent stability of nanodots under a physiological environment [102, 103]. Their particle size of about 5 nm allowed for effective accumulation in tumors [102, 103]. By reacting with water, the created CuO_2_ nanodots sparked a chemical change that produced hydrogen peroxide, and the presence of Cu^2+^ as catalysts sparked a Fenton-like process that produced the very reactive hydroxyl radicals with hydrogen peroxide acting as the reactant on its own [104]. By causing lysosomal lipid peroxidation, the generated hydroxyl radicals caused cancer cells to undergo cell death by lysosomal membrane permeabilization [105, 106].

CaO_2_ nanoparticles should be combined with other Fenton compounds in order to achieve therapeutic goals since the chemically inert Calcium portion cannot cause chemical reactions [107]. With the help of hyaluronate acid, CaO_2_ nanoparticles were combined with widely studied and highly biocompatible Fe_3_O_4_ Fenton nanoagents to create CaO_2_-Fe_3_O_4_/HA hybrid nanostructure, which led to hydrogen peroxide self-supply and Fenton-based tumor killing process [100].

Chemodynamic therapy is a new nanotheranostic method that uses a meticulously synthesized Fenton nanocatalyst to accelerate the conversion of hydrogen peroxide to OH [108, 109]. The impact of chemodynamic therapy is generally inadequate because it is restricted by the quantity of endogenous hydrogen peroxide in the tumor [106, 110]. Since metal peroxides can produce hydrogen peroxide in the mildly acidic TME, it can be used to improve chemodynamic therapy effectiveness. Furthermore, the metal ions that make up metal peroxides, such as Cu^2+^, Co^2+^, and Mn^2+^, have strong Fenton catalytic performance, rendering metal peroxide a prospective hydrogen peroxide self-supply chemodynamic therapy agent [111].

Several researchers have reported Fenton-type copper peroxide (CP) nanodots that were attached by PVP using hydroxide ions [100, 112–115]. As discussed in the abovementioned paragraph, in an acidic condition, the produced CP nanodots may reversibly degrade into Cu^2+^ and hydrogen peroxide, allowing the hydrogen peroxide self-supplying chemodynamic therapy to be produced. The pH-sensitive CP nanodots were absorbed by tumors due to improved permeation and retainment properties, and they produce huge quantities of OH in the acidic endo/lysosomal compartments via a Fenton-like process, which can cause lysosomal membrane permeabilization-mediated tumor cell death via lysosomal lipid peroxidation [37, 106, 113]. Finally, researchers used inductively coupled plasma optical emission spectrometry to examine the physiological dispersion of CP nanopods in U87MG tumor-bearing mice, finding that tumor absorption of CP nano pods was 5.96 0.79 percent, with outstanding chemodynamic therapy antitumor efficacy and minimal loss in weight [113].

The Fenton reaction has been widely employed in water treatment studies since it was first described [116]. In general, the interaction between Fe^2+^ and H_2_O_2_ might result in •OH, which could then destroy the water contaminants [117]. For the Fenton reaction to function properly in industrial settings, a number of parameters, such as the high demand for H_2_O_2_ and maintaining a small optimal pH window, are crucial. Researchers have shown that the Fenton reaction can cause oxidative damage to the cancer cells' DNA, proteins, or lipids, which can be targeted for treatment [118]. The right conditions are created for the Fenton reaction (Fe^2+^ + H_2_O_2_ ⟶ Fe3^+^ + •OH + OH−) to take place by the overexpression of H_2_O_2_ (100 M) and moderate acidity of TME [119].

Designing Fe-based nanosystems for targeted intracellular Fenton reaction with noninvasive therapy effectiveness makes sense given the extremely short half-life of •OH (109 s) [120]. Other transition metal ions, such as Mo^4+^, Ti^3+^, Cu^+^, Mn^2+^, Ag^+^, and V^2+^ have been included in the construction of many nanosystems and nanozymes to help further ease the small window of acidic pH required for effective cancer CDT [46]. Cu^+^ may, for instance, carry out Fenton-like reactions up to 160 times more quickly than Fe^2+^ and is said to be more effective in producing toxic •OH in TME (pH 6.5–6.9) [121]. These Fenton-like reactions caused by transition metals have a number of benefits, including excellent performance in nearly neutral environments and a large natural abundance of structurally diverse oxide products [122].

Fe-based nanocatalysts require low pH levels and large catalyst dosages, but in contrast to other species, they have the best activity at low H_2_O_2_ concentrations and low activation energies [123]. Before precisely designing a Fenton/Fenton-like reaction-based nanomedicine, it is important to take into account the feasibility of active redox cycles in the pH state, catalyst loading, and stability of oxidation products. The full potential of chemodynamic cancer therapy is frequently limited by the intricacy of TME and the preparation of an “all-in-one” chemodynamic drug [124]. Designing appropriate Fenton nanosystems and modifying TME in favour of CDT is therefore of utmost importance.

According to certain theories, ROS trigger intracellular lipid peroxidation, which results in ferroptosis [125] as illustrated in Figure 6. However, treatment is challenging due to the tiny levels of produced OH in cells [126]. There have been reports of several nanoparticles that improve the efficacy of Fenton reactions for medicinal applications [95].

Typically made primarily of metal ions and peroxo groups, metal peroxides may combine with water to form hydrogen peroxide (H_2_O_2_). There are several biological uses for the postgenerated H_2_O_2_. For instance, in catalytic medicine, H_2_O_2_ can function as the reactant in a Fenton-like catalytic reaction to produce enormous amounts of hydroxyl radicals (•OH) [127]. Additionally, H_2_O_2_ has the ability to self-decompose to create oxygen (O_2_), which may be used to increase the therapeutic effectiveness of other O_2_-involved modalities including radiation treatment and photodynamic therapy (PDT). In order to produce O_2_ and H_2_O_2_, metal peroxide can therefore serve as a solid precursor [33]. With a high level of tumor selectivity, Fenton reaction-based catalytic nanotherapeutics have become a unique tumor-therapeutic technique [128].

The development of MO_2_ as a self-supplying source of O_2_ and H_2_O_2_ (Figures 7 and 8) has made it a very promising therapeutic treatment for tumors [129]. Under acidic circumstances, the produced H_2_O_2_ from MO_2_ reacting with H_2_O not only causes oxidative stress but also generates additional O_2_ by serving as a reaction substrate for molecules like CAT or MnO_2_ to reduce tumor hypoxia and reverse TME [130].

### 3.1. Reactive Oxygen Species in Apoptosis

Superoxide radicals (O_2_^−^), singlet oxygen (^1^O_2_), hydrogen peroxide, and hydroxyl radicals are examples of reactive oxygen species (ROS) that may damage lipids, proteins, and DNA, causing cell death and apoptosis. Oxidative stress occurs when ROS levels surpass the antioxidant capability of cells, resulting in cell death [131, 132]. Metal peroxides are excellent in inducing oxidative stress in cells, and it has been widely employed in anticancer therapy in recent times. The mildly acidic tumor microenvironment is expected to break down MO_2_ into M^2+^ and hydrogen peroxide.

Several researchers have reported the synthesis of transferrin-modified MgO_2_ nanosheets (TMNSs), which have a similar reaction to the neutral pH and low CAT activity of the tumor microenvironment [133, 134]. MgO_2_ interacts with H+ to produce hydrogen peroxide quickly, damaging the morphology of transferrin on the nanosheets' surface [135]. The trapped Fe^3+^ is then released by transferrin, which causes the Fenton reaction to produce cytotoxic Hydroxyl radicals [98, 136].

Figure 9 is a Jablonski diagram showing the mechanism of photodynamic cancer therapy mediated by photosensitizers. Photodynamic therapy uses photosensitizers (PS) to transform local molecular oxygen into cytotoxic reactive oxygen species (ROS), which can destroy biomolecules and cause cell death [137, 138]. However, because photodynamic therapy's efficacy is highly dependent on oxygen levels, solid tumor hypoxia reduces its efficacy, and increased oxygen consumption by photodynamic therapy would exacerbate the tumor's hypoxia, creating a vicious cycle [139]. Metal peroxides act as an oxygen self-sufficient compound which improves the effect of the aforesaid challenges of photodynamic therapy.

Zhang et al., for example, created a double light-driven photodynamic therapy using a liposome-based nanosystem [140]. The hydrophilic PS (methylene blue, MB) and CaO_2_ NPs were enclosed in the aqueous cavity and the hydrophobic layer, respectively. When LipoMB/CaO_2_ reaches the tumor tissue, the CaO_2_ inside the liposomes reacts with water to produce oxygen in the mildly acidic TME, alleviating tumor hypoxia [141].

During the first phase, brief irradiation is used to rupture the liposome by oxidizing the phospholipid bilayer and to activate singlet oxygen (^1^O_2_) [141, 142]. CaO_2_ is then exposed to water and generates additional oxygen. Finally, after irradiation is supplied, the photodynamic therapy impact will be much enhanced in the oxygen-adequate TME. This well-conceived two-stage irradiation method based on CaO_2_ maximizes CaO_2_'s oxygen supply capability.

Self-supplying oxygen photodynamic therapy treatment using CaO_2_ and hydrophilic ammonium bicarbonate (NH_4_HCO_3_) encapsulated in PEG-shelled liposomes has also been described using aza Boron-dipyrromethene (BODIPY) dye as photosensitizer (Figure 10) [143]. NH_4_HCO_3_ is used as a thermoresponsive compound in this experiment. Aza BODIPY dye raises the temperature of the liposome system when it is treated with near-infrared (NIR) [143]. When the temperature reaches 40 degree Celsius, NH_4_CO_3_ thermally decomposes to form CO_2_, which expands and destroys the liposomes, enabling CaO_2_ and CO_2_ to completely react to release oxygen, and enhancing the photodynamic therapy effectiveness [143].

Photodynamic therapy using rose bengal as PS was developed with the aid of CaO_2_ NPs and it achieved the best results in these tests [144, 145].

### 3.2. Improved Chemodynamic Therapy

Chemodynamic therapy (CDT) is a developing, minimally invasive technique, which disproportionates endogenous H_2_O_2_ via Fenton or Fenton-like processes into the highly toxic hydroxyl radical (•OH) [95]. By destroying DNA, inactivating proteins, and inducing phospholipid membrane peroxidation, •OH can induce a significant extent of cell death in cancerous cells [146]. CDT is selective since it works well under increased production of hydrogen peroxide in tumors relative to normal tissue. This minimizes the harm to normal tissue. Therefore, compared to conventional treatment options, CDT has a number of benefits, including low invasiveness, excellent selectivity, and fewer adverse effects.

The endogenous concentration of H_2_O_2_ is 10–50 *μ*M [147]. However, this level is inadequate to produce enough hydroxyl radicals to ensure that CDT works effectively. Therefore, the creation of new techniques that will raise the level of H_2_O_2_ in the tumor will raise the level of hydroxyl radical produced by Fenton or processes that are similar to Fenton, which will boost the effects of CDT [148].

The utilization of biochemical processes is one such method to raise the endogenous levels of H_2_O_2_ in tumors [149]. Enzyme catalysis is the major method used for this [150]. Two biological processes have been employed recently to produce H_2_O_2_ in tumors. First, glucose oxidase (GO_*x*_) is used to accelerate the reaction of water, oxygen, and glucose to form gluconic acid and H_2_O_2_ [151]. The alternative process uses superoxide dismutase (SOD) to catalyse the production of H_2_O_2_ from superoxide anion radicals [150]. Both processes create H_2_O_2_ by catalytic reactions using chemicals found in the tumor, which can effectively raise the H_2_O_2_ content.

Metal peroxide can create oxygen or function as a reaction substrate to counteract tumor hypoxia and provide more oxygen for chemo-drugs to deliver improved chemotherapeutic treatment [100]. Due to the limited negative effects, they have on normal tissues *in vivo*, metal peroxides which are broken down by the acidic microenvironment of the tumor to produce metal ions and H_2_O_2_ are a credible alternative source of H_2_O_2_ [129]. In response to the acidic tumor microenvironment, the transferrin-modified MgO_2_ nanosheets rapidly generate a substantial amount of H_2_O_2_ and then undergo a Fenton reaction with metal released from transferrin, which substantially enhanced the production of toxic •OH for the effective cancer therapy [152].

MnO_2_ nanoparticles have been investigated as a smart chemodynamic approach to improve CDT in cancer therapy. After being taken up by the cell, MnO_2_ can interact with intracellular GSH to form GSSG and Mn^2+^, which has good Fenton-like activity when it comes to producing highly reactive hydroxyl radicals from endogenous H_2_O_2_ in the presence of physiological HCO_3_^−^ ions.  Figure 11 shows a scheme of how GSH depletion impairs the antioxidant defence system (ADS), making cancer cells more susceptible to OH radicals produced in the Mn^2+^-mediated Fenton-like process, permitting increased CDT leading to cell death [153].

## 4. Targeting Metal Ion Homeostasis

So far, only a few forms of metal peroxide have been described for tumor treatment, with the majority of the studies focusing on CaO_2_-based nanostructures [154, 155]. Other metal peroxide-based nanoparticles, such as MgO_2_, BaO_2_, ZnO_2_, and CuO_2_-based materials, have yet to be fully realized, and their physiological uses are equally restricted [44]. Improving them by correctly altering them or coupling them with other chemotherapeutic drugs might be a potential research trend [156]. CaO_2_ has the highest clinical translation value in the metal peroxide indicated above, in our opinion. CaO_2_ has strong biocompatibility because Ca^2+^ is extensively dispersed in the body [157].

Furthermore, because Ca^2+^ is dispersed throughout cancer cells, therapy tactics such as calcium stress are universal, and Ca^2+^ has the function of speeding osteogenesis, which might be beneficial in the management of bone cancers such as osteosarcoma [158]. However, the synthesis and preservation of CaO_2_ and metal peroxide face difficulties due to their instability; the shape, size, and dispersion of metal peroxide are hard to accurately regulate, making mass synthesis challenging [34, 159].

Calcium excess is triggered by a malfunction of the calcium balancing system and a problem of calcium transport, which results in an excessive rise in intracellular calcium levels [160, 161]. Calcium excess can disrupt the mitochondrial oxidative phosphorylation pathway, reduce mitochondrial membrane potential, and activate phospholipases and proteases in the cytoplasm, resulting in permanent cell damage [162]. Internal calcification is commonly detected in some cancers following radiation or chemotherapy in clinical treatment, therefore calcification is typically thought of as a byproduct of tumor treatment, and it has been discovered that calcified tumors often respond better to treatment [163, 164].

Given the significance of Ca^2+^ in cell growth, respiration and mortality, the overload mechanism might be destructive to cancerous cells, providing a drug-free approach to cancer treatment [164]. Signal transmission in cells is a fundamental and crucial aspect of life. Ca^2+^ is a broadly distributed intracellular messenger where it regulates nearly all cellular functions in cells, including muscular movement, neurotransmission from neurons and astrocytes, tissue repair, and respiratory functions in the liver and pancreas, together with cellular mitosis, maturity, and death, among others. Ca^2+^ regulates the growth of cancerous cells, tumor progression, invasion, and spread, among other things [164].

Under typical conditions, cells have a very stringent Ca^2+^ level regulation system. However, in an oxidatively stressed environment, cells struggle to maintain Ca^2+^ balance due to aberrant intracellular Ca^2+^ channel activity, culminating in calcium excess-induced cell death [165]. As a result, one of the probable approaches for antitumor treatment is the disruption of tumor physiological Ca^2+^ balance by calcium overload [166].

An oxidatively stressed environment will alter the protein functions and prevent the proper relay of the calcium signal in CAT-downregulated cancerous cells, resulting in unrestrained Ca^2+^ build-up and cell death [167, 168]. Similarly, nanosystems which used CaO_2_ as an oxygen source and hematoporphyrin monomethyl as a photosensitizer have been synthesized and reported [169, 170]. This approach effectively coupled photodynamic therapy with calcium overload.

Cancer cells can also be destroyed by disrupting intracellular Zn^2+^ homeostasis, where ZnO, ZnO_2_, and other Zn-based nanoparticles that may release Zn^2+^ at tumor locations have been studied for tumor treatment [45, 171]. Excess Zn^2+^ can cause apoptotic cell death and lactate dehydrogenase release by depolarizing mitochondrial membrane potential, activating caspase-3, and causing cell death [172]. Simultaneously, by blocking the mitochondrial electron transport chain, Zn^2+^ can boost the production of endogenous ROS [173, 174]. As a result, for Ca^2+^ or Zn^2+^ ion antitumor treatment, the design and synthesis of degradable nanoparticles containing these ions hold great promise.

The produced hydrogen peroxide combines with Fenton or Fenton-like compounds (such as Fe^2+^, Mn^2+^, Cu+, and Co^2+^) to form hydroxyl radicals and achieve chemodynamic therapy in an acidic environment [127, 175]. The hydrogen peroxide generated can be degraded by CAT or MnO_2_ to generate oxygen, enhancing the efficiency of oxygen-dependent cancer treatments such as photodynamic therapy and radiation treatment [176, 177].

The metal ions released after the degradation are observed to have some significant ramifications, such as excess calcium caused by Ca^2+^ ions released from CaO_2_ which is thought to cause mitochondrial damage [166, 178, 179]. The released Ba^2+^ ions produced by the degradation reaction of BaO_2_ are known to act as a potassium ion pump suppressor, inhibiting tumor progression [180, 181].

## 5. Combination Therapies

Even though it is currently a highly popular treatment option for many different types of cancer, monotherapy is usually thought to be less efficient than combination therapy. Traditional monotherapy approaches nonselectively target cells that are actively multiplying, which eventually results in the death of both malignant and healthy cells.

For the majority of cancers, the treatment's effectiveness with monotherapy is insufficient and therefore essential to combine two or even more treatment approaches [182, 183]. Each therapeutic drug has antitumor action, and by combining them, they can provide the effects of combination therapy. Additionally, the “1 + 1 > 2” synergistic therapeutic outcomes can be achieved if the tumor-killing mechanisms of each therapeutic drug can complement one another [184].

More significantly, the properties of metal peroxides may be precisely paired with photosensitizers, enzymes, metal nanoparticles, Fenton reagents, or chemotherapeutic medications, among other things, to help and encourage different therapies including photodynamic therapy, chemodynamic therapy, and chemotherapy [170, 185, 186]. When several therapies are coupled, metal peroxide-based coadministration achieves much better antiproliferative results [187].

Because metal peroxides are unstable, some surface modification using molecules such as polyvinyl pyrrolidone (PVP) and hyaluronic acid (HA) is required for improved biological applications in physiological media [188, 189]. Surface modification enhances not only the stability of metal peroxide but also the dispersibility of nanoparticles (NPs), making tumor targeting feasible [190, 191].

A key component of cancer therapy is combination therapy, a mode of care that combines two or more therapeutic drugs. The combination of anticancer medications improves efficacy in comparison to monotherapy because it targets important pathways in a manner that is often additive or synergistic [192]. In addition to therapeutic anticancer effects including reducing tumor growth and metastatic potential, this strategy may also diminish drug resistance [79]. Being able to target several pathways effectively reduces drug resistance because cancer cells typically cannot adapt to the concurrent harmful effects of two therapeutic drugs. The process of creating a new anticancer medicine is expensive and time-consuming. New tactics are thus being proposed that focus on survival routes that deliver efficient and effective outcomes at a reasonable cost.

Combination therapy with drugs originally prescribed for the management of conditions other than cancer is one such strategy. In the end, this has a synergistic or cumulative effect, necessitating a smaller therapeutic dosage of each drug, because they enable the use of individual medications in lower dosages while maintaining therapeutic efficiency. These combination drug regimens lessen the overall toxicity of the treatment.

This strategy works best when an FDA-approved medication targets pathways that are comparable to those seen in cancer [193]. The overall cost of combination treatment research is decreased because one of the medications utilized in it is already FDA-approved [194]. The various outcomes from monotherapies and combination therapies are summarized in Figure 12.

Traditional cancer treatments generally only destroy differentiated cancer cells and miss the cancer stem cells (CSC). Thus, CSC is capable of surviving and may cause relapses. CSC-targeted medicines either eradicate CSC or cause differentiation in cancer cells, which may then lead to apoptosis-mediated cell death. However, combined therapy may be the most successful method of removing tumors.

## 6. Synthetic Procedures for Metal Peroxides

The most extensively used process for preparing metal peroxides is hydrolyzation-precipitation [100, 195]. Metal chloride, metal acetate, or metal carbonate are commonly utilized as precursors in this process, which involves adding hydrogen peroxide to an alkaline aqueous medium of metal salt to precipitate the water-insoluble metal peroxide particles [196]. The procedure is relatively simple and is carried out under mild conditions making the process to be cheap, and the size of NPs may be controlled to several nanometres.

For example, in the synthesis of CaO_2_, the CaO_2_ hydrate was formed using equation (1) and the process was subsequently aided in precipitating the metal peroxide by adding ammonia to neutralize the HCl, as shown [196, 197]:

(1) $$\begin{array}{c} {CaCl}_{2}+hydrogen\;peroxide+2HCl⟶{CaO}_{2}\left(hydrate\right) \end{array}$$

It is important to note that, in addition to regulating the size of the particles, PVP also works as a stabilizer in hydrolyzed precipitation [35, 198]. The synthesis of BaO_2_ by hydrolysis and precipitation process described the use of PEG as a stabilization agent to change the outer layer of metal peroxide [199].

In a nutshell, sodium formate and BaCl_2_ aqueous solution were ultrasonically combined before being added to dry methanol. After aggressively swirling, hydrogen peroxide is added to the mixture, and the BaO_2_ NPs were precipitated using an aqueous solution of choline hydroxide [200].

They noted that the organic ligands used had a significant impact on the growth rate and orientation of BaO_2_ nanocrystals, resulting in a variety of sizes of particles and morphologies. When a ligand with a specified coordination capacity with Ba^2+^ is added to the process, the crystal development is successfully regulated, resulting in nanosized BaO_2_ particles [200]. Nanoparticles with varied particular surface areas and functionalities have varied shape controllability, which is an important link in the design of nanoparticle theranostic platforms. To limit the toxicity of free Ba^2+^ to healthy tissue, the scientists combined BaO_2_ with a biodegradable potent chelating ligand L-glutamic acid (N-diacetic acid) in the abovementioned illustration [200]. Effective surface modification not only enhances the stability of metal peroxide but also the dispersion of NPs, making tumor targeting possible.

The Leidenfrost dynamic chemistry approach is another synthetic option. Here in this method, the formation and development of NPs are split into the following two sections: initially, nanochemistry happens in the heated zone, and the generated NPs create nanoclusters; secondly, these nanoclusters move into cooler regions, where they will continue to grow [200, 201]. This propensity might be used to control the size of NPs in the future. Zinc acetate solution was combined with hydrogen peroxide and put in a Petri dish, which was then rapidly exposed to a superheated plate (300 C), causing the solution to change colour from colourless to milky white, resulting in the formation of ZnO_2_ NPs [200, 201]. Overall, by adjusting the concentration of zinc acetate, the size of ZnO_2_ NPs produced by this approach could be controlled.

Literature reports on the production of MgO_2_ nanosheets have been published via a microemulsion system, where cyclohexane and CO-5_2_0 were added to an MgCl_2_ solution [200, 202–204]. After 30 minutes of stirring, ammonium hydroxide was quickly introduced to generate Mg(OH)_2_ and stirred for another 30 minutes. To generate MgO_2_ nanosheets, hydrogen peroxide was introduced to regulate the reaction process, and anhydrous ethanol was used to break the reverse microemulsion system [200]. Similarly, a reverse microemulsion approach to synthesize CaO_2_ nanoparticles by simultaneously incorporating cisplatin, and capping with negatively charged phospholipid has been reported [205, 206].

The sizes of NPs may be controlled in a microemulsion process by altering the moisture content and pH of the micelles [207, 208]. In the microemulsion process, the organic solvent layer and surfactant layer efficiently separated the precipitated particles and increased particle dispersibility [209, 210]. Some chemotherapy medications can be introduced directly to the microemulsion system to create NPs while also achieving drug loading [205].

The ideal approach for the research study on the biomimetic production of calcium carbonate (CaCO_3_) minerals is the gas diffusion technique, which has the benefits of ease of operation and monitoring [94, 211]. Deng and coworkers devised a new CaO_2_ production method based on CaCO_3_ gas diffusion chemistry. A beaker with ethanol solution with CaCl_2_ and hydrogen peroxide is typically covered with parafilm with some holes, and then another separate beaker holding ammonia is then introduced in the same desiccator. The CaO_2_ synthesis is completed after a 2-hour gas diffusion process at 35°C [212].

ZnO_2_ nanoparticles have been produced via an innovative sonochemical method [213, 214]. The method is a straightforward reaction where ZnSO_4_H_2_O was dissolved in distilled water and NaOH was added dropwise to adjust the pH up to 8.0 [213]. After that, hydrogen peroxide was added, and the mixture was sonicated with ultrasound for half an hour, yielding ZnO_2_ nanoparticles with very uniform size ranges and a spherical shape [213]. However, nanoparticle aggregation was detected. The best way to modify size distribution and optimize NP distribution has never been straightforward [215]. Metal peroxide has been used as an oxygen-generating compound in the production of potential tumor theranostics nanoplatforms in the past few years, which may modulate the tumor microenvironment to generate a new working environment for therapies whose effectiveness is restricted by the underlying tumor microenvironment [44, 46, 213, 215, 216].

## 7. Conclusion

Even if there are still many issues to be resolved, metal peroxides have introduced innovative methods for treating tumors, and their use in biology merits further research and development. Metal peroxide nanostructures have been produced and applied as a supply of oxygen and hydrogen peroxide in the cancer tumor microenvironment with promising results [100]. Under acidic environments, the hydrogen peroxide produced by the reaction of metal peroxide with water has a dual role of inducing oxidative stress and producing surplus oxygen from the reaction with molecules such as catalyse enzymes. These alleviate tumor hypoxia thereby reversing the low oxygen levels observed in the tumor microenvironment [29, 216, 217]. In addition, the properties of metal peroxides may be precisely paired with other molecules such as photosensitizers, enzymes, metal nanoparticles, Fenton reagents, or chemotherapeutic medications, to achieve combination therapies including photodynamic therapy, chemodynamic therapy, and chemotherapy [170, 185–187]. Metal peroxide-based coadministration with other therapies has been shown to achieve much better antiproliferative results [187].

Though not exhaustive, this review visited the most widely studied metal peroxide nanosystems that have been applied in cancer studies. It covers common synthesis procedures for these nanomaterials and a comprehensive overview of applications in the noncellular cancer tumor microenvironment.

## Figures and Tables

**Figure 1:** Estimated percentage of deaths from various cancers in the US in 2021.

**Figure 2:** Applications for various metal peroxide nanotherapeutics.

**Figure 3:** Approaches for targeting the tumor microenvironment.

**Figure 4:** Mechanism of hypoxia-activated AQ4N and enamine N-oxide prodrugs.

**Figure 5:** Summary mechanism of tripazamine under normal and hypoxic cells.

**Figure 6:** Mechanism of ROS generation by ferroptosis.

**Figure 7:** Fenton chemistry of MO_2_ as a self-supplying source of O_2_ and H_2_O_2_.

**Figure 8:** Mechanism of catalytic chemistry of Fenton nanocatalysts for versatile radical nanotherapeutics.

**Figure 9:** Mechanism of photosensitizer-mediated photodynamic cancer therapy.

**Figure 10:** Two-stage mechanism of CaO_2_ and boron aza BODIPY photodynamic therapy.

**Figure 11:** Cancer treatment through nanoparticle-facilitated Fenton process.

**Figure 12:** Comparison of the effectiveness of traditional monotherapies and combination therapies.

## Data Availability

All data used to support this study are included within the article.
